# Diffuse Uterine Leiomyomatosis: A Rare Case of Symmetrically Enlarged Uterus

This article has been retracted.

**DOI:** 10.7759/cureus.60827

**Published:** 2024-05-22

**Authors:** Divyajat Kumar, Vishav Bir S Thakur, Suhas M

**Affiliations:** 1 Department of Radiodiagnosis, Dr. D. Y. Patil Medical College, Hospital & Research Centre, Dr. D. Y. Patil Vidyapeeth (Deemed to Be University), Pune, IND

**Keywords:** primary infertility, nullipara, uterine mass, multiple leiomyoma, diffuse uterine leiomyomatosis

## Abstract

A rarely reported case of diffuse uterine leiomyomatosis is observed in a 43-year-old nulliparous female presenting with abdominal distension and primary infertility. Magnetic resonance imaging (MRI) of the abdomen and pelvis revealed an enlarged uterus with multiple well-defined lobulated lesions of varying sizes, causing symmetrical uterine enlargement and displacing the adjacent bowel loops superolaterally. The compression of the bladder and inferior vena cava was seen without the involvement of the adjacent structures. The diagnosis of diffuse leiomyomatosis of the uterus was confirmed through histopathological examination of the biopsy.

## Introduction

Leiomyomas, also known as benign fibroids, represent smooth muscle tumours found in the uterus. They affect approximately 25% of women during their reproductive years. While the exact cause of these growths remains incompletely understood, their frequent occurrence in premenopausal women and their tendency to regress after menopause indicate a probable hormonal influence [1]. Another type of smooth muscle tumour affecting the uterus is diffuse uterine leiomyomatosis (DUL), also considered a neoplastic condition [2]. This rare disorder is characterised by symmetric enlargement of the uterus, primarily due to numerous ill-defined and merged nodules almost completely replacing the uterine myometrium [3].

Less than 50 cases have been documented in the literature. The initial case, documented by Murray and Glynn in 1924 under the term 'complete uterine fibromyomatosis', was later reclassified as 'diffuse uterine leiomyomatosis' by Lapan and Solomon in 1979 [4]. Baschinsky et al. observed that different tumour sites within DUL originated from distinct clonal lineages, supporting the concept of independent neoplastic origins. They proposed that DUL might represent an extreme manifestation of multiple uterine leiomyomas merging into one another and blending seamlessly, making individual nodules indiscernible upon gross examination [1]. The nodules seamlessly integrate with one another and blend indistinguishably into the surrounding myometrium, which is comparatively less cellular and normal. Microscopic analysis reveals that the nodules consist of densely packed fascicles and intertwined bundles of benign smooth muscle cells [5].

The primary symptoms at the onset of DUL typically comprise abdominal discomfort and irregular uterine bleeding. These initial presentations may manifest as menorrhagia, dysmenorrhoea, abdominal pain, infertility, and pelvic pressure, which are similar to the symptoms seen in leiomyomas [1,3]. Typically, clinical manifestations of the condition arise between the third and fourth decades of life, when patients may express a desire for future pregnancy. Hormonal therapies often prove ineffective in managing symptoms, anaemia, or tumour growth cessation once the treatment is stopped [6]. Patients receiving hormonal treatment or undergoing minimally invasive hysteroscopic myomectomy have reported successful pregnancies. Additional therapeutic approaches encompass uterine artery embolisation, high-intensity focused ultrasound (HIFU), and sirolimus administration [7].

Our report describes DUL in a 43-year-old nulliparous woman who presented with primary infertility as her chief complaint. The case highlights radiological findings and histopathological features associated with DUL.

## Case presentation

A 43-year-old nullipara, seeking conception, presented to the obstetrics and gynaecology outpatient department due to primary infertility following two years of marriage. Despite one year of unprotected intercourse, she had not achieved pregnancy and sought medical evaluation for infertility. The patient had a history of menarche at the age of 12 years, with regular menstrual cycles lasting 25 days and menstrual bleeding lasting four to five days. She denied experiencing dyspareunia, menorrhagia, metrorrhagia, or dysmenorrhoea. There were no remarkable findings in the patient's past medical, family, or surgical history, nor in her history of allergies or contraceptive use. Physical, systemic, and breast examinations revealed no significant findings except for minimal abdominal distension, predominantly on the right side. Palpation revealed a large, firm mass with a smooth surface and regular margins, extending from the pubic symphysis to the epigastric region. The mass demonstrated restricted mobility, and there was limited access to its lower margins in the pelvis. The speculum examination showed normal findings, except for a superiorly displaced mobile cervix with fullness in the lateral fornices. A radiological examination was recommended for further evaluation.

On ultrasound examination, the abdominopelvic mass was confirmed to be an enlarged uterus with numerous hypoechoic masses of variable sizes. These masses showed increased vascularity on the colour Doppler scale and filled the entire uterine myometrium. The patient subsequently underwent magnetic resonance imaging (MRI) of the abdomen and pelvis to further characterise these findings. A contrast-enhanced MRI of the pelvis revealed a grossly enlarged uterus measuring 24 x 11 x 22 cm in maximum dimensions. Multiple well-defined lobulated lesions of varying sizes (ranging from 1.5 to 5.5 cm) were diffusely involved throughout the entire myometrium. These lesions appeared hypointense on T1-weighted images (Figure 1) and heterogeneously hypointense to isointense on T2-weighted images with intervening hyperintense areas (Figure 2). Additionally, a few areas exhibited diffusion restriction (Figure 3). The lesions were predominantly intramural, with a few subserosal lesions replacing the uterine myometrium.

**Figure 1:** The coronal section of the abdomen and pelvis in T2-weighted imaging shows a grossly enlarged uterus with multiple T2 heterogenous signal intensity intramural fibroids (red block arrows), leading to extensively thickened uterine myometrium (3 Tesla MRI). MRI: magnetic resonance imaging.

**Figure 2:** Multiple heterogeneous intensity lesions are showing diffusion restriction (red stars) on DWI (A) with corresponding low ADC values (B) (red line arrows) on magnetic resonance imaging (3 Tesla MRI). MRI: magnetic resonance imaging; DWI: diffusion-weighted imaging; ADC: apparent diffusion coefficient.

**Figure 3:** The axial section of the abdomen and pelvis in T2-weighted imaging shows a grossly enlarged uterus with multiple T2 heterogenous signal intensity intramural fibroids (red block arrows) in the lower uterine segment (3 Tesla MRI). MRI: magnetic resonance imaging.

The enlarged uterus exerted a mass effect, displacing the abdominal bowel superoposteriorly, compressing the bladder inferiorly, and pushing the inferior vena cava (IVC) posteriorly without loss of fat planes or involvement of the adjacent structures. The endometrium was displaced, measuring 7 mm in thickness, while the ovaries were displaced laterally. No cystic changes were visualised, and the nodules demonstrated relatively homogeneous enhancement on the T1-weighted post-gadolinium sequences on the MRI of the pelvis (Figure 4). A differential diagnosis of multiple leiomyomas was considered, with the primary possibility being diffuse leiomyomatosis of the uterus.

**Figure 4:** The coronal section of the pelvis in T1-weighted post-contrast imaging shows no significant enhancement of the lesions (red block arrows) filling the entire uterine myometrium (3 Tesla MRI). MRI: magnetic resonance imaging.

The patient received a detailed explanation of her current condition, including management options and potential outcomes. Subsequently, a diagnostic hysteroscopy was performed to obtain a tissue biopsy sample, revealing benign neoplastic changes in the smooth muscle cells upon histopathological examination (Figure 5). Following confirmation of the benign nature of the lesion, the patient was referred to the obstetrics and gynaecology department for further management, with multiple myomectomy chosen to preserve fertility. Unfortunately, she was unable to follow up due to affordability issues regarding surgery.

**Figure 5:** Histopathological examination of the biopsy with hematoxylin & eosin stain (H&E). (A) Original magnification x 10—the slide under the microscope shows intersecting fascicles on hematoxylin & eosin stain (H&E); (B) original magnification x 40—oval to spindle-shaped cells having vesicular to hyperchromatic nuclei and scant-to-moderate eosinophilic cytoplasm. No atypical mitosis was seen.

## Discussion

DUL is classified as a benign neoplasm originating from the uterine myometrium, yet its precise aetiology remains unknown. Limited understanding of this condition stems from its infrequent documentation in the medical literature [4]. It is characterised by the presence of numerous, indistinct [8] and typically small-sized leiomyomas with a few centimetres in diameter, which extensively involve the entire myometrium, resulting in symmetric enlargement of the uterus. It primarily affects women in the later stages of their reproductive years, often presenting with symptoms such as menorrhagia and infertility [1,9].

Risk factors for diffuse leiomyomatosis include being a female of African-American descent in the reproductive age group and having a family history of uterine leiomyomas. However, the specific risk factors directly linked to diffuse leiomyomatosis have not been established, although there is an association with Alport syndrome. Alport syndrome predominantly exhibits X-linked inheritance in approximately 85% of cases, with around 5% of affected individuals demonstrating diffuse leiomyomatosis involving the female genital tract, oesophagus, and tracheobronchial tree [10].

Ultrasonography serves as the primary imaging modality for evaluating pelvic, uterine, and ovarian conditions. Early detection of DUL is challenging, often leading to misdiagnosis prior to surgical intervention due to the absence of distinct manifestations [11]. MRI is often considered the modality of choice for evaluating the female pelvis due to its ability to provide multiplanar imaging and excellent contrast for soft tissues. Additionally, MRI plays a crucial role in pre-treatment planning by offering comprehensive mapping, including assessment of the number, size, and location of leiomyomas within the uterine layers, as well as aiding in differential diagnosis [12]. Diagnosis relies heavily on preoperative MRI and postoperative histopathological examination. Currently, there is no standardised diagnostic approach for the condition. MRI plays a crucial role in early detection and comprehensive preoperative assessment [4]. Diffuse leiomyomatosis on MRI mimics its gross pathological appearance. On radiological imaging, the uterus shows characteristic symmetrical enlargement due to near-complete replacement by innumerable, mostly small-sized leiomyomas with indistinct margins, merging together with coalescing fibres, giving a "pebble-filled purse" appearance [5,8]. This differs from cases of multiple leiomyomas, which are typically well-defined nodules with a pseudocapsule causing asymmetrical involvement and distortion of the uterus [1]. Individually, leiomyomas on T2-weighted images show low to intermediate signal intensity as compared to normal myometrium. However, this difference is not distinctly appreciated in diffuse leiomyomatosis due to near-complete myometrial replacement. Contrast-enhanced T1-weighted images reveal variable enhancement patterns of the uterine masses [8]. Leiomyomas can be found submucosally, intramurally, or subserosally in both of these conditions. In our case, they are well appreciated in the intramural region.

The widespread involvement of the uterine myometrium in diffuse leiomyomatosis can make it challenging to identify individual leiomyomas, rendering a complete myomectomy unattainable. In cases of incomplete myomectomy, there is a risk of symptom recurrence in the future due to the inability to excise all lesions individually. Consequently, hysterectomy has been established as the standard therapeutic approach for diffuse leiomyomatosis, particularly in individuals who no longer wish to maintain fertility [13].

Certain disorders are considered in the differential diagnosis of DUL, which include the following: (a) diffuse uterine adenomyosis and (b) diffuse endometrial hypertrophy can be distinguished through histopathological examination. DUL differs from (c) multiple leiomyomas in that the latter shows asymmetrical uterine involvement with well-defined masses, while multiple leiomyomas show uniform and symmetrical involvement of the entire myometrium by smooth muscle nodules with poorly defined borders and merging masses [14]. (d) Disseminated peritoneal leiomyomatosis is characterised by multiple mature smooth muscle nodules affecting the mesentery, visceral, and parietal fascia of the peritoneum, often coexisting with uterine leiomyomas [15]. (e) Uterine lymphangiomyomatosis is distinguished by the invasion of pulmonary vascular spaces [15]. (f) Intravascular leiomyomatosis presents with worm-like intravascular smooth muscle extensions, which have a creamy to yellow appearance and reveal the presence of some or all neoplastic smooth muscles with vascular channels [14]. Other differential diagnoses include (g) hereditary leiomyomatosis and renal cell carcinoma (HLRCC) [4], (h) Alport syndrome with diffuse leiomyomatosis (ASDL) [4], and (i) endometrial stromal sarcoma [14].

Literature reports instances of successful pregnancies in women undergoing treatment with gonadotropin-releasing hormone agonists or minimally invasive hysteroscopic myomectomy for the removal of submucosal leiomyomas [8,16]. Another conservative method showing encouraging outcomes is uterine artery embolisation (UAE). Currently, UAE is being extensively used for the management of symptomatic fibroids and is gaining widespread recognition as an effective substitute for hysterectomy or myomectomy. Consequently, it merits consideration as a treatment option for reproductive-aged women with diffuse leiomyomatosis [16], whereas hysterectomy has been established as the prevailing therapeutic strategy for diffuse leiomyomatosis, especially in individuals who no longer intend to preserve fertility [4].

## Conclusions

DUL has an unknown aetiology and is often misdiagnosed due to its rarity and limited literature. It is typically diagnosed after a histopathological examination of the hysterectomy specimen. An MRI of the pelvis plays an important role in diagnosis and preoperative assessment. While hormonal therapies often provide temporary relief, recurrence following conservative surgery has been documented. Consequently, hysterectomy remains the final option, even for younger patients in the later stages of their reproductive lives.

In conclusion, MRI plays a crucial role in reliably diagnosing diffuse leiomyomatosis, allowing for the best possible approach to its management based on the patient's desired level of fertility. Therefore, radiologists need to be well-versed in this benign condition and its imaging characteristics.
